The article "LncRNA TP73-AS1 down-regulates miR-139-3p to promote retinoblastoma cell proliferation" was published in 2019. Journal: Biosci Rep.

# LncRNA TP73-AS1 down-regulates *miR-139-3p* to promote retinoblastoma cell proliferation

**DOI:** 10.1042/BSR20190475

**Published:** 2019-05-10

**Authors:** Zhaoxia Xia, Xiaoxi Yang, Shuduan Wu, Zhizhen Feng, Lei Qu, Xianghua Chen, Linyu Liu, Yanling Ma

**Affiliations:** Department of Opthalmology, The Sixth Affiliated Hospital of SUN Yat-sen University, Guangzhou City, Guangdong Province 510655, PR. China

**Keywords:** lncRNA TP73-AS1, miR-139-3p, proliferation, retinoblastoma

## Abstract

Our study aimed to investigate the role of long non-coding RNAs (lncRNA) TP73-AS1 in retinoblastoma (Rb). In the present study, we found that TP73-AS1 was up-regulated, while *miR-139–3p* was down-regulated in Rb. TP73-AS1 and *miR-139-3p* were inversely correlated in Rb tissues. In cells of Rb cell lines, overexpression of *miR-139-3p* failed to affect TP73-AS1, while TP73-AS1 overexpression caused the down-regulated *miR-139-3p*. TP73-AS1 overexpression caused promoted proliferation of Rb cells but showed no significant effects on cell migration and invasion. *miR-139-3p* overexpression played an opposite role and attenuated the effects of TP73-AS1 overexpression. Therefore, lncRNA TP73-AS1 may down-regulate *miR-139-3p* to promote Rb cell proliferation.

## Introduction

Retinoblastoma (Rb) is a common and deadly intraocular tumor that mainly affects children [1]. Incidence of Rb is relatively low comparing to other types of malignancy. Only one out of 18000 to 30000 live births will develop Rb worldwide [2]. However, without proper treatment, development of Rb is rapid and brain metastasis is common, leading to high mortality rate [3]. Based on international Classification of Rb, patients with Rb can be classified into A–E groups. Chemotherapy is usually successful in the treatment of group A–C patients, while ocular survival rate of group D after systemic chemotherapy is only 10–47% [4]. In addition, this rate in group E patients is close to 0 [5,6]. Therefore, novel therapeutic targets are always needed.

Many factors, such as age, gender and laterality affect the occurrence and development of Rb, while genetic alterations are the key determinants in this process [7,8]. Besides oncogenes and tumor suppressors that participate in cancer biology by producing functional proteins, non-coding RNAs (ncRNAs), such as long (>200 nt) ncRNAs (lncRNAs) also have an important roles in cancer development and progression by regulating gene expression [9,10]. LncRNA TP73-AS1 has been characterized as an oncogenic lncRNA in many types of cancers, such as osteosarcoma and glioma [11,12]. Our preliminary deep sequencing data revealed an inverse correlation between TP73-AS1 and *miR-139-3p*. A recent study reported that *miR-139-3p* inhibited cancer cell invasion, migration and proliferation in glioma [13], while its involvement in Rb is unclear. The present study was carried out to study the role of TP73-AS1 and *miR-139-3p* in Rb and to explore the interactions between them.

## Materials and methods

### Patients and specimens

Our study enrolled 56 patients with Rb (31 males and 25 females, 1.1–4.9 years, 2.6 ± 0.5 years). All those patients were admitted by The Sixth Affiliated Hospital of SUN Yat-sen University during the time period between September 2016 and October 2018. All those patients were diagnosed by histopathological biopsy. Patients received any therapies before admission, patients failed to cooperate with researchers, patients complicated with other clinical disorders or patients with a previous history of malignancies were excluded from the present study. According to the International Classification for Intraocular Retinoblastoma, there were 11, 16, 10, 12 and 7 cases at group A–E, respectively. All patients signed informed consent. Ethics Committee of aforementioned hospital approved the present study before the admission of patients.

Rb (cancer) and non-cancer (2 cm around tumors) tissues were obtained from each patient through biopsy. All tissue specimens were confirmed by at least four pathologists.

### Cells and transient transfections

WERI-Rb-1 and Y79 two human Rb cell lines were used. Cells of both cell lines were from ATCC (U.S.A.). RPMI-1640 Medium (20% FBS) was used as the cell culture medium. Cell culture conditions were 37°C and 5% CO_2_.

TP73-AS1 expression vector was constructed by inserting full length TP73-AS1 cDNA into pcDNA3.1 vector (Sangon, Shanghai, China). Negative control (NC) miRNA and *miR-139-3p* mimic were from Sigma–Aldrich (U.S.A.). Before transfection, WERI-Rb-1 and Y79 cells were cultivated overnight to reach 70–80% confluence. After that, 10 nM vectors or 40 nM miRNAs were transfected into WERI-Rb-1 and Y79 cells through Nucleofector™ Technology. Subsequent experiments were performed at 24 h after transfections. Cells without transfections (Control) and cells transfected with NC miRNA or empty vector were included to serve as two controls.

### RT-qPCR

Ribozol (Thermo Fisher Scientific., lnc.) was used to extract total RNAs from tissue specimens as well as WERI-Rb-1 and Y79 cells. Following cDNA synthesis using AMV Reverse Transcriptase XL (Clontech, U.S.A.), qPCR reaction systems were prepared using SYBR Green Master Mix (Bio-Rad, U.S.A.) to detect the expression of TP73-AS1. MiRNA extractions were extracted from tissue specimens as well as WERI-Rb-1 and Y79 cells using mirVana miRNA Isolation Kit (Thermo Fisher Scientific., lnc.). Following reverse transcriptions using TaqMan MicroRNA Reverse Transcription Kit (Thermo Fisher Scientific., lnc.), qPCR reaction systems were prepared using Applied Biosystems™ TaqMan™ MicroRNA Assay (Thermo Fisher Scientific) to detect the expression of *miR-139-3p* with U6 as endogenous control. All qPCR reactions were performed three times and data were processed using 2^−ΔΔ*C*^_T_ method. The sample with the lowest Δ*C*_T_ value was set to “1” and all other samples were normalized to this sample.

### Measurement of Rb cell proliferation rate

WERI-Rb-1 and Y79 cells were harvested at 24 h after transfections to prepare single cell suspensions using RPMI-1640 Medium (20% FBS), and cell density was adjusted to 3 × 10^4^ cells per ml. Single cell suspensions were transferred to a 96-well plate (0.1 ml per well). Cells were cultivated at 37°C with 5% CO_2_, and CCK-8 solution (10 μl, Sigma–Aldrich, U.S.A.) was added every 24 h until 96 h after the beginning of cell culture. Cells were then cultivated for further 4 h, followed by the addition of 10 μl DMSO. Finally, OD values at 450 nm were measured.

### Statistical process

Experiments were repeated three times to obtain solid experimental data. Differences between Rb and non-cancer tissues were analyzed by paired *t*-test. Differences among different disease groups or among different groups of cell transfections were analyzed by one-way ANOVA and Tukey *t*-test. Linear regression was performed to analyze the correlation between TP73-AS1 and *miR-139-3p*. Differences were statistically significant when *P*<0.05.

## Results

### TP73-AS1 and m*iR-139-3p* were dysregulated in Rb tissues

Expression of TP73-AS1 and *miR-139-3p* was detected by performing RT-qPCR, followed by analysis of the expression data by paired *t*-test. It was found that TP73-AS1 was significantly up-regulated (Figure 1A, *P*<0.05), while *miR-139-3p* was significantly down-regulated (Figure 1B, *P*<0.05) in Rb tissues than in non-cancer tissues of Rb patients, indicating the involvement of TP73-AS1 and *miR-139-3p* in Rb.

**Figure 1:** TP73-AS1 and *miR-139-3p* were dysregulated in Rb tissues Analysis of TP73-AS1 and *miR-139-3p* expression data showed that TP73-AS1 was significantly up-regulated (**A**), while *miR-139-3p* was significantly down-regulated (**B**) in Rb tissues than in non-cancer tissues of Rb patients (*P<0.05).

### TP73-AS1 and *miR-139-3p* were affected by the development of Rb

According to International Classification for Intraocular Retinoblastoma, there were 11, 16, 10, 12 and 7 cases at group A–E, respectively. Expression data of TP73-AS1 and *miR-139-3p* were compared among different groups by performed one-way ANOVA and Tukey test. It was found that expression levels of TP73-AS1 increased (Figure 2A), while expression levels of *miR-139-3p* decreased (Figure 2B) with the development of Rb (*P*<0.05).

**Figure 2:** TP73-AS1 and miR-139-3p were affected by the development of Rb Analysis of TP73-AS1 and *miR-139-3p* analysis by one-way ANOVA and Tukey test showed that expression levels of TP73-AS1 increased (**A**), while expression levels of *miR-139-3p* decreased (**B**) with the development of Rb. Group A, tumor size below 3 mm, not lose to foveola or optic disc, only in the retina; Group B, tumor larger than 3 mm, close to foveola or optic disc, only in the retina; Group C, small amounts of spread into the jelly-like material or under the retina; Group D, subretinal seeding or widespread vitreous; Group E, large tumor extends near the front of the eye, glaucoma or bleeding, (*P<0.05).

### TP73-AS1 and *miR-139-3p* were inversely correlated

Linear regression was performed to analyze the correlation between TP73-AS1 and *miR-139-3p*. A significant and reverse correlation between TP73-AS1 and *miR-139-3p* was found in Rb tissues (Figure 3A), but not in non-cancer tissues (Figure 3B).

**Figure 3:** TP73-AS1 and *miR-139-3p* were inversely correlated Linear regression revealed a significant and reverse correlation between TP73-AS1 and *miR-139-3p* was found in Rb tissues (**A**), but not in non-cancer tissues (**B**).

### TP73-AS1 down-regulated *miR-139-3p* to promote the proliferation of Rb cells

To further explore the interactions between TP73-AS1 and *miR-139-3p*, TP73-AS1 expression vector or *miR-139-3p* mimic were transfected into WERI-Rb-1 and Y79 cells. Comparing to C (Control) and NC (Negative control), expression levels of TP73-AS1 and *miR-139-3p* were significantly up-regulated at 24 h after transfection (Figure 4A, *P*<0.05). Comparing to the two controls, overexpression of *miR-139-3p* failed to affect TP73-AS1 (Figure 4B), while TP73-AS1 overexpression caused down-regulated *miR-139-3p* (Figure 4C, *P*<0.05). Analysis of cell proliferation data showed that TP73-AS1 overexpression caused promoted proliferation of both WERI-Rb-1 and Y79 cells (Figure 4D, *P*<0.05), but showed no significant effects on cell migration and invasion (data not shown, revealed by the data of Transwell migration and invasion assay). In addition, *miR-139-3p* overexpression played an opposite role and attenuated the effects of TP73-AS1 overexpression (*P*<0.05).

**Figure 4:** TP73-AS1 down-regulated *miR-139-3p* to promote the proliferation of Rb cells Comparing to C (Control) and NC (Negative control), expression levels of TP73-AS1 and *miR-139-3p* were significantly up-regulated at 24 h after transfection (**A**). Comparing to the two controls, overexpression of *miR-139-3p* failed to affect TP73-AS1 (**B**), while TP73-AS1 overexpression caused down-regulated *miR-139-3p* (**C**). Moreover, TP73-AS1 overexpression caused promoted proliferation of both WERI-Rb-1 and Y79 cells (**D**). In addition, *miR-139-3p* overexpression played an opposite role and attenuated the effects of TP73-AS1 overexpression (^*^P<0.05).

## Discussion

The present study investigated the involvement of TP73-AS1 in Rb and explored its functions in this disease. We showed that TP73-AS1 was up-regulated in Rb and promoted Rb cell proliferation by down-regulating *miR-139-3p*, which has been characterized as a tumor suppressive miRNA in Rb [13].

We observed that TP73-AS1 was up-regulated in many types of cancers, and regulated cancer cell behaviors to promote cancer development [11,12]. Therefore, TP73-AS1 may also have the same expression pattern and functions in Rb. The present study showed that TP73-AS1 was up-regulated in Rb and its expression level increased with the development of Rb, which confirmed our hypothesis. TP73-AS1 participates in cancer biology through the interactions with multiple downstream cancer-related pathways, such as HMGB1/RAGE pathway in both glioma and liver cancer [12,14]. However, we did not observe the interaction between TP73-AS1 and HMGB1/RAGE pathway in Rb cells (data not shown, revealed by Western blot after TP73-AS1 overexpression). Therefore, TP73-AS1 may play its oncogenic roles by interacting with different signaling pathways in different types of malignancies.

Previous studies reported the interactions between TP73-AS1 and miRNAs in cancer biology, such as the down-regulation of tumor suppressive *miR-124* and *miR-200a* by TP73-AS1 in glioma and breast cancer, respectively [15,16]. TP73-AS1 serves as a sponge of these miRNAs [15,16]. Our study proved that TP73-AS1 was likely an upstream inhibitor of *miR-139-3p* in the regulation of Rb cell proliferation. Interestingly, miR-139-3p inhibits cancer cell migration and invasion in different types of cancers including Rb [13,17]. However, TP73-AS1 overexpression resulted in down-regulated mR-139-3p in Rb cells but failed to affect cancer cell migration and invasion. This is possibly due to the specific cell lines used in the present study. Another explanation is that mR-139-3p is already down-regulated in Rb and the further down-regulation of mR-139-3p by TP73-AS1 overexpression may not be reflected by cancer cell migration and invasion. It is worth noting that expression levels of *miR-139-3p* varied a lot across non-cancer tissues. Therefore, *miR-139-3p* expression may be also regulated by certain factors other than Rb, such as patients’ habits and genetic background. Our future studies will perform deeper analyses.

The present study investigated the role of TP73-AS1 in regulating Rb cell proliferation. In addition, TP73-AS1 may not affect Rb cell migration and invasion. However, its roles in regulating other behaviors of Rb cells, such as cell cycle progression and cell apoptosis are unknown. In glioma it is known that TP73-AS1 affects the expression of p53 to regulate cancer cell apoptosis. Our future studies will explore the functions of TP73-AS1 in regulating other behaviors of Rb cells. In conclusion, TP73-AS1 was up-regulated in Rb and TP73-AS1 overexpression may down-regulate mR-139-3p to promote Rb cell proliferation.

## Availability of data and materials

The analyzed datasets generated during the study are available from the corresponding author on reasonable request.

## Abbreviations

lncRNA: long non-coding RNA
NC: negative control
ncRNAs: non-coding RNA
Rb: retinoblastoma
